# Genetic variation in the leukotriene pathway is associated with myocardial infarction in the Chinese population

**DOI:** 10.1186/s12944-019-0968-9

**Published:** 2019-01-24

**Authors:** Yilan Li, Xueming Xu, Dandan Zhang, Wei Cheng, Yanan Zhang, Bo Yu, Yao Zhang

**Affiliations:** 1 Department of Cardiology, the 2nd Affiliated Hospital of Harbin Medical University, Harbin, 150001 China; 2 Key Laboratory of Myocardial Ischemia, Ministry of Education, Harbin Medical University, Harbin, 150001 China; 3 Department of Cardiology, Heilongjiang Provincial Hospital, Harbin, 150001 China

**Keywords:** Arachidonate 5-lipoxygenase, Arachidonate 5-lipoxygenase-activating protein, Single nucleotide polymorphism, Myocardial infarction, Coronary artery disease

## Abstract

**Background:**

Genetic variation in the genes ALOX5 (arachidonate 5-lipoxygenase), ALOX5AP (arachidonate 5-lipoxygenase-activating protein) and LTA4H (leukotriene A4 hydrolase) has previously been shown to contribute to the risk of MI (myocardial infarction) in Caucasian and African American populations. All genes encode proteins playing a role in the synthesis of the pro-inflammatory leukotriene B mediators, possibly providing a link between MI and inflammation. The aim of the present study was to investigate whether these associations could be confirmed in the study of China MI patients. The study included 401 Han Chinese MI patients and 409 controls. Six tag single nucleotide polymorphisms (SNPs)—ALOX5 rs12762303 and rs12264801, ALOX5AP rs10507391, LTA4H rs2072512, rs2540487 and rs2540477—were selected. SNP genotyping was performed by an improved multiplex ligation detection reaction assay.

**Results:**

The rs2540487 genotype was associated with the risk of MI in overdominant model (*P* = 0.008). rs12762303 and rs10507391 SNPs were significantly associated with lipid levels in MI patients (*P* < 0.006–0.008). Several SNPs interacted with alcohol consumption, cigarette smoking, and hypertension to modify TC, TG, LDL-C and CRE levels, and the risk of MI (*P* < 0.0017 for all). No association between the SNPs of LT pathway and susceptibility to MI was found (*P* > 0.05 for all).

**Conclusions:**

Taken together, this study provides additional evidence that functional genetic variation of the LT pathway can mediate atherogenic processes and the risk of MI in Chinese.

## Background

Coronary artery disease (CAD), and its most severe complication myocardial infarction(MI), are leading causes of death and disability worldwide [1, 2]. Multiple factors, including genetic, environmental, and psychological factors, were believed to contribute to the onset of CAD [3]. A plethora of evidence has demonstrated that atherosclerosis is a major pathologic change in CAD, and inflammatory reactions and immune function disorders are implicated in the development of CAD [4, 5]. In recent years, focus has turned on the complex cascade of inflammatory processes that takes place in the vessel wall and within atherosclerotic plaques [6–8]. In this context the leukotriene pathway has received attention.

The initial enzymatic step in the leukotriene pathway is the oxidation of arachidonic acid to leukotriene A4 (LTA4) by 5-lipoxygenase (5-LO, encoded by ALOX5) [9]. A necessary cofactor in this reaction is the 5-lipoxygenase-activating protein (FLAP), encoded by the arachidonate 5-lipoxygenase-activating protein (ALOX5AP) gene, is an important mediator of the activity of 5-lipoxygenase, a key enzyme in the biosynthesis of leukotrienes [10]. The LTA4H gene encodes leukotriene A4 hydrolase, a protein in the same biochemical pathway as ALOX5AP [11]. LTA4 is further hydrolyzed by leukotriene A4 hydrolase (LTA4H) to leukotriene B4 (LTB4) or conjugated to produce a series of three related to cysteinyl leukotrienes (LTC4, LTD4, LTE4) by the LTC4 synthase (LTC4S) enzyme [12]. LTs are thought to be potent chemotactic molecules that mediate the recruitment of neutrophils, monocytes, and other leukocytes to sites of inflammation, including the arterial wall of atherosclerotic lesions [13, 14] (Fig. 1).

**Fig. 1:** The activation of 5-lipoxygenase (5-LO) pathway of AA metabolism by the enzymes 5-lipoxygenase activating protein (FLAP) and 5-lipoxygenase (5-LO) will catalyze the conversion of AA into the chemokine, leukotriene A4 (LTA4), which will be converted into other leukotrienes by the enzymes LTA4 hydrolase (LTA4H) and LTC4 synthase (LTC4S). These leukotrienes act on leukotriene receptors in lymphocytes, endothelial, and smooth muscle cells, which further enhance inflammatory reactions and subsequently, atherogenesis

Despite the accumulating evidence linking the 5-LO pathway to atherosclerosis, no Chinese genetic studies have substantiated a relationship between LT pathway polymorphisms and clinical complications of atherosclerosis including MI [10]. Several genetic linkage and associations studies as well as gene expression studies have shown an association of the ALOX5/ALOX5AP pathway to CAD. This stems from a series of biochemical, genetic, and pharmacological studies over the last few years that have provided evidence for the pro-atherogenic role of LTs [14, 15]. For example, genetic deficiency for ALOX5 in mice increases mortality after MI because of healing defects [16]. This is not mediated by a change in local blood flow, but through an altered inflammation and/or fibroblast function. Other mouse studies have reported the involvement of LT pathway genes in atherosclerosis related traits as well, including the LT receptors and ALOX5 activating protein (ALOX5AP) [17, 18].

The leukotriene pathway has been implicated in the pathogenesis of cardiovascular but the detailed mechanistic basis for their pathophysiological roles is still a matter of discussion. Moreover, none of the previous studies specifically attempted to dissect the role of LT pathway in the atherosclerosis phenotype rather than in its ‘complication’ phenotype (MI) [19]. The goal of this study was therefore to comprehensively evaluate the genetic contribution of the LT pathway in individuals with MI. Such information may have the potential to provide predictive value for assessing cardiovascular risk [12].

## Results

### General characteristics of the subjects

Table 1 compares the general characteristics and lipid levels between the patients and controls. The population included in the study comprises a total of 810 individuals. As illustrated, the majority of study participants are male (82.0%), about two-third are current smokers (60.3%), and 26.2% drinking alcohol. The mean age, gender distribution, hypercholesterolemia and triglycerides level were not different between controls and MI patients (*P* > 0.05 for all). With the exception of hypercholesterolemia and triglycerides, the risk factors generally occurred more frequently among the cases than the controls. (*p* < 0.05 for all).

**Table 1:** Baseline characteristics of the study participants

Variables	MI (*n* = 401)	Controls (*n* = 409)	*P*-value^a^
Age, years	58.20 (11.65)	56.34 (9.52)	0.223
Male sex, No. (%)	329 (82.0%)	339 (82.9%)	0.753
Smoking, No. (%)	242 (60.3%)	187 (45.7%)	**3.04E-05**
Alcohol, No. (%)	105 (26.2%)	82 (20.0%)	**0.038**
Diabetes, No. (%)	99 (26.7%)	50 (12.2%)	**4.71E-06**
Hypertension, No. (%)	192 (47.9%)	143 (35.0%)	**1.90E-4**
Hypercholesterolemia, No. (%)	55 (13.7%)	39 (9.5%)	0.063
WBC, 10^9^/L	11.96 (3.81)	6.84 (1.90)	**1.78E-80**
FBG, mmol/L	7.13 (3.86)	5.93 (1.93)	**1.25E-7**
CRE, μmol/L	85.67 (30.17)	70.83 (13.30)	**3.22E-18**
AST, U/L	80.44 (85.24)	25.12 (9.43)	**2.54E-32**
Total cholesterol, mmol/L	4.56 (1.05)	4.96 (0.84)	**7.03E-9**
Triglycerides, mmol/L	1.65 (1.12)	1.67 (1.23)	0.764
HDL cholesterol, mmol/L	1.28 (0.43)	1.37 (0.36)	**1.65E-3**
LDL cholesterol, mmol/L	2.77 (0.83)	3.30 (0.73)	**1.92E-20**

Values are means ± SD or n (%). ^a^Two-sided chi-square test or independent-samples *t*-test. ^b^*P*-values < 0.05 are bold. Type 2 diabetes was diagnosed as (1) fasting plasma glucose (FPG) ≥ 7.0 mmol/L; (2) 2 h postprandial glucose ≥11.1 mmol/L; or (3) use of antidiabetes medications. Hypertension was defined as systolic/diastolic blood pressure ≥ 140 mmHg or ≥ 90 mmHg or use of antihypertensive medications. Hypercholesterolemia was defined as use of cholesterol-lowering medications or total serum cholesterol > 200 mg/dl. WBC, white blood cell; FBG, fasting blood glucose; AST, aspartate transaminase; CRE, creatinine; HDL, high-density lipoprotein; LDL, low-density lipoprotein

### Genotypic and allelic frequencies in patients and controls

The genotype and allele frequencies of six SNPs selected for study are shown in Table 2. No deviations from Hardy–Weinberg equilibrium were observed in either cases or controls. The genotype and allele frequencies of the rs12762303, rs12264801, rs10507391, rs2072512, rs2540487, rs2540477 SNPs in MI patients and controls were not significantly different (all *P* > 0.05).

**Table 2:** Genotypic and allelic frequencies of six SNPs in MI patients and controls

SNP/group	Genotype^a^ (n (%))			χ^2^	*P*	Allele		χ^2^	*P*	OR (95% CI)
rs12762303	CC	CT	TT			C	T			
Case	20 (0.05)	111 (0.28)	270 (0.67)			151 (0.19)	651 (0.81)	0.00	0.949	1.01 (0.79–1.29)
Control	18 (0.04)	117 (0.29)	274 (0.67)	1.44	0.23	153 (0.19)	665 (0.81)			
rs12264801	AA	GA	GG			A	G			
Case	86 (0.21)	199 (0.50)	116 (0.29)			371 (0.46)	431 (0.54)	0.45	0.502	0.94 (0.77–1.14)
Control	99 (0.24)	194 (0.47)	116 (0.28)	1.01	0.31	392 (0.48)	426 (0.52)			
rs10507391	AA	TA	TT			A	T			
Case	48 (0.12)	195 (0.49)	158 (0.39)			291 (0.36)	511 (0.64)	0.06	0.805	1.02 (0.84–1.26)
Control	50 (0.12)	192 (0.47)	167 (0.41)	0.21	0.65	292 (0.36)	526 (0.64)			
rs2072512	AA	TA	TT			A	T			
Case	74 (0.18)	180 (0.45)	147 (0.37)			328 (0.41)	474 (0.59)	0.69	0.406	1.08 (0.89–1.33)
Control	68 (0.17)	182 (0.44)	159 (0.39)	1.66	0.20	318 (0.39)	500 (0.61)			
rs2540487	TT	CT	CC			T	C			
Case	25 (0.06)	115 (0.29)	261 (0.65)			165 (0.21)	637 (0.79)	1.82	0.177	0.85 (0.67–1.08)
Control	19 (0.05)	153 (0.37)	237 (0.58)	0.83	0.36	191 (0.23)	627 (0.77)			
rs2540477	GG	GA	AA			G	A			
Case	129 (0.32)	193 (0.48)	79 (0.20)			451 (0.56)	351 (0.44)	0.63	0.426	0.92 (0.75–1.12)
Control	137 (0.33)	202 (0.49)	70 (0.17)	0.09	0.76	476 (0.58)	342 (0.42)			

*SNP* single nucleotide polymorphism, *MI* myocardial infarction

^a^All are in Hardy–Weinberg equilibrium

### Genotypes of the six LT pathway SNPs and the risk of MI

To explore the potential inheritance patterns, four models of inheritance including dominant, recessive, codominant and overdominant models were explored for each SNP (Table 3). The genotype of the LTA4-H rs2540487 was associated with the risk of MI after the Bonferroni correction (a value of *P* < 0.01 was considered statistically significant) in the overdominant genetic model: CC + TT vs. CT (OR = 1.48, 95% CI = 1.11–1.99, *P* = 0.008). Comparison of both heterozygous and homozygous carriers of the minor allele (C) with homozygous carriers of the major allele (T) revealed that the ALOX-5 rs12762303 and rs12264801 SNPs were negatively associated with MI, suggesting a dominant genetic effect. No association of ALOX-5AP rs10507391, LTA4-H rs2072512 or rs2540477 and MI were observed. Similar, but weaker trends were observed for the recessive model, codominant model or overdominant model, with no significant associations of the five SNPs with MI (all *P* > 0.05).

**Table 3:** Genetic model analysis of the association of six SNPs and MI susceptibility

SNP/group	Genotype		χ^2^	*P*	OR (95% CI)
rs12762303					
Dominant	CC+ CT	TT	0.10	0.92	0.98 (0.73–1.32)
Recessive	CC	CT + TT	0.16	0.69	1.14 (0.59–2.18)
Codominant	TT	CT	0.06	0.81	0.96 (0.71–1.31)
		CC	0.12	0.72	1.12 (0.58–2.17)
Overdominant	TT + CC	CT	0.08	0.76	1.04 (0.77–1.42)
rs12264801					
Dominant	AA+GA	GG	0.03	0.85	0.97 (0.72–1.31)
Recessive	AA	GA + GG	0.87	0.35	0.85 (0.61–1.19)
Codominant	GG	GA	0.02	0.88	1.02 (0.74–1.42)
		AA	0.51	0.48	0.87 (0.59–1.28)
Overdominant	GG + AA	GA	0.39	0.53	0.91 (0.70–1.21)
rs10507391					
Dominant	AA +TA	TT	0.17	0.68	1.06 (0.80–1.41)
Recessive	AA	TA + TT	0.12	0.91	0.98 (0.64–1.49)
Codominant	TT	TA	0.22	0.63	1.07 (0.80–1.44)
		AA	0.00	0.95	1.01 (0.64–1.59)
Overdominant	TT + AA	TA	0.23	0.63	0.93 (0.71–1.23)
rs2072512					
Dominant	AA +TA	TT	0.42	0.51	1.10 (0.83–1.46)
Recessive	AA	TA + TT	0.47	0.49	0.79 (1.13)
Codominant	TT	TA	0.18	0.66	1.06 (0.79–1.45)
		AA	0.64	0.42	1.18 (0.79–1.75)
Overdominant	TT + AA	TA	0.01	0.91	0.98 (0.75–1.30)
rs2540487					
Dominant	TT + CT	CC	4.36	0.037	0.73 (0.55–0.98)
Recessive	TT	CT + CC	0.99	0.32	1.36 (0.74–2.51)
Codominant	CC	CT	6.29	0.012	0.68 (0.51–0.92)
		TT	0.31	0.57	1.19 (0.64–2.22)
Overdominant	CC + TT	CT	6.97	**0.008** ^**a**^	1.48 (1.11–1.99)
rs2540477					
Dominant	GG + AG	AA	0.90	0.34	0.84 (0.59–1.20)
Recessive	GG	AG + AA	0.16	0.69	0.94 (0.70–1.26)
Codominant	AA	AG	0.74	0.38	0.85 (0.58–1.23)
		GG	0.78	0.38	0.83 (0.56–1.25)
Overdominant	AA+GG	AG	0.13	0.72	1.05 (0.80–1.39)

SNP, single nucleotide polymorphism; MI, myocardial infarction. A *P* < 0.01 was considered statistically significant after Bonferroni correction. ^a^ *P*-values < 0.01 are bold

### Genotypes and lipid levels

We expected that genetic risk associated with the SNPs would be reflected by established CAD risks, including total cholesterol (TC), triglycerides (TGs), high-density lipoprotein cholesterol (HDL-C), low-density lipoprotein cholesterol (LDL-C), creatinine (CRE), or fasting blood glucose (FBG). As shown in Table 4, the minor C allele of rs12762303was associated with high FBG concentrations in MI patients compared with the control group (*P* = 0.008) and the rs10507391variants were associated with increased TC (*P* = 0.006) after the Bonferroni correction of *P* values. None of the six SNPs were associated with TG, HDL-C, LDL-C or CRE in MI patients (*P* > 0.0083).

**Table 4:** Lipid level and genotype in MI patients and controls

SNP	Genotype (Counts)	TC	TG	HDL-C	LDL-C	CRE	FBG
		mmol/L	mmol/L	mmol/L	mmol/L	μmol/L	mmol/L
rs12762303							
case	TT (270)	4.53 ± 1.13	1.66 ± 1.16	1.28 ± 0.47	2.78 ± 0.86	87.35 ± 31.89	7.36 ± 4.03
	CT (111)	4.63 ± 0.85	1.56 ± 0.79	1.26 ± 0.31	2.76 ± 0.78	82.38 ± 26.64	6.31 ± 3.36
	CC (20)	4.59 ± 0.94	1.93 ± 1.91	1.29 ± 0.33	2.79 ± 0.70	81.25 ± 23.09	8.67 ± 3.29
	*P*	0.718	0.807	0.890	0.936	0.296	**0.008** ^**a**^
control	TT (274)	4.97 ± 0.85	1.71 ± 1.26	1.39 ± 0.40	3.28 ± 0.75	70.82 ± 13.74	6.00 ± 2.05
	CT (117)	4.86 ± 0.88	1.57 ± 1.22	1.36 ± 0.29	3.27 ± 0.73	70.01 ± 12.14	5.81 ± 1.59
	CC (18)	5.13 ± 0.61	1.64 ± 0.72	1.22 ± 0.23	3.39 ± 0.78	76.57 ± 12.84	5.80 ± 1.78
	*P*	0.409	0.134	0.168	0.481	0.063	0.925
rs12264801							
case	AA (86)	4.65 ± 0.96	1.71 ± 1.22	1.27 ± 0.45	2.79 ± 0.89	82.11 ± 25.52	7.47 ± 3.22
	GA (199)	4.57 ± 1.07	1.71 ± 1.18	1.24 ± 0.30	2.75 ± 0.82	88.13 ± 32.29	6.85 ± 4.21
	GG (116)	4.50 ± 1.06	1.49 ± 0.93	1.35 ± 0.57	2.78 ± 0.83	84.09 ± 29.45	7.36 ± 3.65
	*P*	0.737	0.205	0.082	0.990	0.451	0.156
control	AA (99)	4.94 ± 0.77	1.63 ± 1.09	1.31 ± 0.26	3.27 ± 0.76	70.92 ± 13.80	5.91 ± 1.93
	GA (194)	4.99 ± 0.91	1.73 ± 1.40	1.41 ± 0.40	3.30 ± 0.76	71.08 ± 12.52	5.88 ± 1.76
	GG (116)	4.88 ± 0.79	1.58 ± 1.02	1.35 ± 0.37	3.27 ± 0.71	70.38 ± 14.19	6.05 ± 2.16
	*P*	0.253	0.950	0.128	0.891	0.666	0.981
rs10507391							
case	TT (158)	4.77 ± 1.03	1.73 ± 1.30	1.28 ± 0.33	2.85 ± 0.81	81.90 ± 24.50	7.48 ± 3.91
	AT (195)	4.46 ± 1.01	1.64 ± 1.06	1.28 ± 0.51	2.70 ± 0.81	87.82 ± 31.25	7.02 ± 3.81
	AA (48)	4.29 ± 1.15	1.41 ± 0.61	1.23 ± 0.31	2.77 ± 1.00	89.35 ± 40.38	6.44 ± 3.85
	*P*	**0.006**	0.678	0.531	0.165	0.224	0.250
control	TT (167)	4.95 ± 0.93	1.58 ± 1.17	1.35 ± 0.31	3.33 ± 0.80	70.83 ± 12.84	5.87 ± 1.93
	AT (192)	4.93 ± 0.80	1.69 ± 1.21	1.37 ± 0.40	3.24 ± 0.72	70.64 ± 13.95	6.00 ± 2.02
	AA (50)	5.02 ± 0.74	1.84 ± 1.46	1.45 ± 0.40	3.28 ± 0.67	71.68 ± 12.38	5.89 ± 1.45
	*P*	0.708	0.479	0.270	0.677	0.825	0.291
rs2072512							
case	AA (74)	4.64 ± 1.22	1.65 ± 1.11	1.23 ± 0.34	2.83 ± 0.93	92.85 ± 41.31	7.05 ± 4.00
	AT (180)	4.54 ± 1.01	1.57 ± 1.07	1.27 ± 0.32	2.78 ± 0.81	83.11 ± 21.81	7.37 ± 3.79
	TT (147)	4.56 ± 1.00	1.74 ± 1.19	1.31 ± 0.56	2.71 ± 0.81	85.19 ± 31.99	6.89 ± 3.89
	*P*	0.530	0.186	0.847	0.769	0.171	0.504
control	AA (68)	4.88 ± 0.90	1.53 ± 1.17	1.38 ± 0.40	3.22 ± 0.72	69.85 ± 13.40	5.84 ± 2.08
	AT (182)	4.96 ± 0.81	1.67 ± 1.25	1.35 ± 0.30	3.34 ± 0.74	70.49 ± 13.45	5.89 ± 1.95
	TT (159)	4.96 ± 0.86	1.71 ± 1.22	1.40 ± 0.42	3.24 ± 0.77	71.67 ± 13.12	6.03 ± 1.81
	*P*	0.245	0.418	0.809	0.329	0.384	0.343
rs2540487							
case	CC (261)	4.58 ± 1.02	1.70 ± 1.21	1.29 ± 0.45	2.78 ± 0.82	84.94 ± 30.49	7.17 ± 4.09
	CT (115)	4.53 ± 1.11	1.54 ± 0.97	1.29 ± 0.38	2.76 ± 0.89	85.09 ± 27.13	7.19 ± 3.60
	TT (25)	4.52 ± 1.06	1.62 ± 0.73	1.14 ± 0.39	2.69 ± 0.78	96.00 ± 38.53	6.50 ± 2.22
	*P*	0.713	0.530	0.469	0.900	0.166	0.419
control	CC (237)	4.96 ± 0.86	1.70 ± 1.23	1.36 ± 0.35	3.30 ± 0.75	70.82 ± 14.12	6.02 ± 2.00
	CT (153)	4.92 ± 0.83	1.65 ± 1.28	1.38 ± 0.39	3.24 ± 0.72	71.63 ± 11.87	5.84 ± 1.81
	TT (19)	5.01 ± 0.93	1.33 ± 0.71	1.46 ± 0.29	3.32 ± 0.96	64.79 ± 12.61	5.69 ± 1.76
	*P*	0.496	0.484	0.224	0.615	0.161	0.672
rs2540477							
case	AA (79)	4.71 ± 1.20	1.71 ± 1.27	1.23 ± 0.32	2.87 ± 0.91	94.05 ± 38.87	7.04 ± 3.64
	GA (193)	4.54 ± 0.99	1.61 ± 1.14	1.26 ± 0.33	2.76 ± 0.81	80.42 ± 23.65	7.31 ± 3.40
	GG (129)	4.52 ± 1.02	1.66 ± 1.01	1.32 ± 0.58	2.71 ± 0.82	88.39 ± 31.50	6.92 ± 3.80
	*P*	0.367	0.477	0.971	0.508	0.066	0.680
control	AA (70)	4.81 ± 0.85	1.51 ± 1.16	1.34 ± 0.38	3.19 ± 0.71	71.56 ± 13.09	5.91 ± 2.20
	GA (202)	5.03 ± 0.85	1.65 ± 1.21	1.39 ± 0.35	3.35 ± 0.79	69.74 ± 13.54	5.90 ± 1.89
	GG (137)	4.90 ± 0.84	1.77 ± 1.28	1.37 ± 0.38	3.23 ± 0.69	72.10 ± 12.99	6.00 ± 1.81
	*P*	0.073	0.222	0.328	0.154	0.207	0.507

*SNP* single nucleotide polymorphism, *TC* total cholesterol, *TG* triglyceride, *HDL-C* high-density lipoprotein cholesterol, *LDL-C* low density lipoprotein cholesterol, *CRE* creatinine, *FBG* fasting blood glucose. Results are mean ± SD. Significance (*P* < 0.05) was determined by the Kruskal–Wallis test. Significant difference, *P* < 0.0083 after the Bonferroni correction. ^a^*P*-values < 0.0083 are bold

### Interactions of the six SNPs and drinking, smoking, age, sex and hypertension on lipid levels and the risk of MI

The interactions of the six SNPs and drinking, smoking, age, sex and hypertension on lipid levels and the risk of MI are shown in Table 5. The SNP of rs12762303 interacted with alcohol consumption to influence TC level. Several SNPs interacted with age to influence TC (rs12264801 and rs10507391), TG (rs12264801 and rs2540477) and LDL-C (rs10507391) levels. The SNP of rs2540477 interacted with sex to modulate CRE levels. The SNP of rs2540487 interacted with hypertension to influence TG levels.

**Table 5:** The *P* values for interactions of genotypes and age, drinking and smoking, on lipid levels and the risk of CAD

SNP	Factor	TC	TG	HDL-C	LDL-C	CRE	FBG
rs12762303	Drinking	0.022	0.794	0.621	**1.57E-4**	0.883	0.398
	Smoking	0.452	0.633	0.251	0.213	0.721	0.410
	Age	0.084	0.247	0.633	0.162	0.667	0.415
	Sex	0.115	0.560	0.593	0.200	0.050	0.090
	Hypertension	0.863	0.019	0.050	0.077	0.641	0.481
rs12264801	Drinking	0.582	0.549	0.448	0.503	0.747	0.693
	Smoking	0.798	0.528	0.163	0.838	0.669	0.666
	Age	**5.21E-4** ^**a**^	**3.47E-4**	0.500	0.010	0.071	0.530
	Sex	0.282	0.642	0.110	0.622	0.003	0.003
	Hypertension	0.418	0.006	0.033	0.813	0.135	0.164
rs10507391	Drinking	0.916	0.728	0.633	0.236	0.595	0.961
	Smoking	0.899	0.299	0.082	0.465	0.631	0.803
	Age	**1.92E-4**	0.006	0.706	**2.83E-4**	0.321	0.924
	Sex	0.307	0.847	0.090	0.778	0.023	0.034
	Hypertension	0.570	0.038	0.260	0.864	0.044	0.337
rs2072512	Drinking	0.361	0.962	0.629	0.639	0.436	0.915
	Smoking	0.396	0.095	0.240	0.932	0.671	0.259
	Age	0.016	0.012	0.391	0.010	0.051	0.033
	Sex	0.460	0.402	0.505	0.784	0.011	0.019
	Hypertension	0.114	0.002	0.157	0.457	0.930	0.348
rs2540487	Drinking	0.150	0.359	0.988	0.020	0.678	0.941
	Smoking	0.878	0.478	0.174	0.281	0.054	0.468
	Age	0.018	0.010	0.912	0.079	0.178	0.998
	Sex	0.808	0.457	0.900	0.432	0.517	0.191
	Hypertension	0.031	**0.001**	0.191	0.546	0.261	0.150
rs2540477	Drinking	0.787	0.763	0.898	0.229	0.717	0.926
	Smoking	0.777	0.110	0.147	0.787	0.609	0.533
	Age	0.010	**8.73E-6**	0.320	0.069	0.095	0.312
	Sex	0.367	0.811	0.228	0.771	**0.001**	0.071
	Hypertension	0.049	0.002	0.210	0.533	0.677	0.064

*SNP* single nucleotide polymorphism, *TC* total cholesterol, *TG* triglyceride, *HDL-C* high-density lipoprotein cholesterol, *LDL-C* low-density lipoprotein cholesterol, *FBG* fasting blood glucose, *CRE* creatinine, *MI* myocardial infarction. Significant difference, *P* < 0.0017 after the Bonferroni correction. ^a^*P*-values < 0.0017 are bold

## Discussion

Recent LT pathway studies of MI have discovered multiple gene locus. However, most of the studies have focused on samples of non- Asian origin, and the identified loci altogether explain only a small fraction of the risk for MI. Moreover, the variants identified in these populations descent might not be applicable in Chinese because of underlying genetic heterogeneity. Therefore, larger scale studies in Chinese are needed to reveal new susceptibility loci and improve our understanding of LT pathway to MI. This study identified interactions between gene polymorphisms in leukotriene production enzymes and the clinical complications of atherosclerosis mainly about MI in Chinese Hans [20].

Our study showed that ALOX5 rs12762303 was associated with fasting blood glucose (FBG) levels but not with MI in Chinese population, which is consistent with the studies by Assimes et al. [10]. A recent study by Mehrabian et al. demonstrated that Alox5−/− mice had significantly increased fat mass, plasma leptin levels and fasting glucose levels, but lower fasting insulin levels [21]. These results provide strong evidence for pleiotropic metabolic effects of 5-LO on adiposity and pancreatic function and may have important implications for therapeutic strategies targeting this pathway for the treatment of cardiovascular disease.

Our study showed that ALOX5AP rs10507391 was associated with total cholesterol (TC) levels but we didn’t observe any association between rs10507391 and the risk of MI. This is in line with the findings of Guoping et al. [22], who found a consistent no association of acute coronary syndrome with the A allele of the same polymorphism. Moreover, ALOX5AP has been previously associated with atherosclerosis [15], whereas its haplotypes have been associated with myocardial infarction [11].

The most significant association detected in our discovery sample set was between a SNP of LTA4H (rs2540487) and MI subjects assuming an overdominant model of inheritance. The potential effects of polymorphisms in rs2540487 upon the development of coronary atherosclerosis or acute MI have not been well studied. To the best of our knowledge, there have been no prior studies examining whether rs2540487 polymorphisms are associated with acute MI or with CAD. We found the genotype of rs2540487 was significantly different between MI and control group by overdominant model analysis (*P* = 0.008, OR = 1.48, 95% CI = 1.11–1.99). It indicates that homozygotes of rs2540487 are more suitable than heterozygotes for MI in Chinese Han population. In addition to classical risk factors genetic predisposition may thus play an important role in the pathogenesis of MI in Chinese Han population.

We found no convincing association between SNPs in ALOX5 (rs12264801) or LTA4H (rs2072512 and rs2540477) and MI. Previous human genetic study concerning the relationship of rs2540477 polymorphism with CAD have yielded inconsistent results [13]. Jaana Hartiala et al. have reported a significant association between rs2540477 and CAD with the T allele being risky. Moreover, they have demonstrated that also haplotype HapK, containing this T allele, results in an increased risk for CAD [13]. In spite of the above-reviewed positive findings, there are other studies that failed to demonstrate this type of associations for CAD or MI, including a case–control study nested within the Multi-Ethnic Study of Atherosclerosis Cohort in the US [23], a case-cohort study in Denmark [24], and a US study that recruited participants mostly from young adults [10]. The lack of consistent findings among the published studies could be due to differences in allelic and haplotype frequency of underlying causal variants and extent of LD between causal and non-causal variants in different populations [25].

Several limitations should be acknowledged in the present study. First, the sample size was relatively small and the participants were limited to Chinese ethnicity. Second, there were differences in some clinical characteristics between the patients and controls. Although several confounders have been adjusted for the statistical analyses, we could not completely eliminate the potential influences of these factors on the results. Finally, the biological mechanism of genetic variants about the LT pathway were not conducted in this study. Larger studies should be followed up to assess the potential association of the SNPs with more complex, clinical-disease-related endpoints.

## Conclusion

In conclusion, the six SNPs in the leukotriene pathway were not associated with the risk of MI in this Han Chinese population, although MI patient characteristics were affected by gene polymorphisms. The results of the present study showed that the rs2540487 genotype was associated with the risk of MI in overdominant model. Those with rs12762303CC genotype had higher FBG levels than those with rs12762303TT and rs12762303CT genotypes. Those with rs10507391TT genotype had higher TC levels than those with rs12762303AA and rs12762303AT genotypes. Several SNPs interacted with alcohol consumption, cigarette smoking and hypertension to modify TC, TG, LDL-C and CRE levels, and the risk of MI. However, this study was designed as a pilot study and further investigations are needed to confirm our results and to elucidate unresolved questions. The contribution of other genetic variants of these vascular-related genes to CAD and MI cannot be excluded.

## Methods

### Sample collection

A total of 401 hospitalized MI patients were enrolled at the Second Affiliated Hospital, Harbin Medical University (China) between September 2016 and November 2017. The study protocol was approved by the local ethics review board; all participants provided written informed consent. MI was diagnosed by symptoms within 24 h of hospital admission, an electrocardiogram consistent with MI, and positive troponin-I. Patients with recent illnesses or infections were not eligible [26]. A group of 409 age- (5-year bands) and sex-matched medical center patients without a history of CAD or symptoms of MI were selected as controls. Patients with cerebrovascular, neurological, or kidney disease, blood disorders, cancer, peripheral vascular disease, or autoimmune diseases were excluded from the control group. Participant age, sex, blood pressure, lipid profile, fasting glucose, medical, drug, smoking, and alcohol histories were collected.

### SNP selection

Four leukotriene pathway loci were selected by a tagSNP method using Haploview version 4.2 bioinformatics software (Broad Institute, Cambridge, MA, USA; https://www.broadinstitute.org/haploview/haploview) assuming a minor allele frequency > 0.05 and a squared correlation between genotypes (푟^2^) > 0.8 for the SNPs in the Han Chinese population (CHB + CHS). The SNP information was retrieved from the 1000 Genomes Project database (http://browser.1000genomes.org) and included those associated with cardiovascular disease in recent studies.

### DNA extraction and genotyping

The genomic DNA was extracted using a GeneJET Whole Blood Genomic DNA Purification Mini Kit (Thermo Scientific, USA) as per the product instruction. The SNP genotyping work was performed using an improved multiplex ligation detection reaction (iMLDR) technique developed by Genesky Biotechnologies Inc. (Shanghai, China). A multiplex PCR-ligase detection reaction method was used in the iMLDR. For each SNP, the alleles were distinguished by different fluorescent labels of allele-specific oligonucleotide probe pairs. Different SNPs were further distinguished by different extended lengths at the 3’end. Two negative controls were set: one with double-distilled water as template and the other with DNA sample without primers while keeping all other conditions the same in one plate. Duplicate tests were designed and the results were consistent. A random sample accounting for ~ 5% (*n* = 40) of the total DNA samples was directly sequenced using Big Dye-terminator version 3.1 and an ABI3730XL automated sequencer (Applied Biosystems) to confirm the results of iMLDR.

### Statistical analyses

All statistical analyses were performed using SPSS 13.0 (SPSS Inc., Chicago, IL, USA) and Microsoft Excel 2016 (Microsoft Corp., Redmond, WA, USA). All tests were two-sided and *P*-values < 0.05 were considered significant. Between-group differences in demographic characteristics and genotype frequencies of the six SNPs were evaluated by Student’s *t*-test for continuous variables and χ2 tests for categorical variables. The Hardy–Weinberg equilibrium was assessed for controls using the goodness-of-fit χ2 test. Associations of genotypes and alleles and the risk of MI were estimated by odds ratios (ORs) and 95% confidence intervals (CIs). The association between genotypes and lipid parameters was tested by analysis of covariance (ANCOVA). Any variants associated with the lipid parameter at a value of *P* < 0.0083 (corresponding to *P* < 0.05 after adjusting for six independent tests by the Bonferroni correction) were considered statistically significant. Significant interactions of the six SNPs with alcohol consumption, cigarette smoking, age, sex, and hypertension with lipid levels and the risk of MI were detected by the independent-samples *t*-test for categorical variables and linear regression analysis for continuous variables after controlling for potential confounders, a *P*-value < < 0.0017 after the Bonferroni correction was considered statistically significant.

## Abbreviations

ALOX5: Arachidonate 5-lipoxygenase
ALOXAP: Arachidonate 5-lipoxygenase-activating protein
CAD: Coronary artery disease
LTA4H: Leukotriene A4 hydrolase
MI: Myocardial infarction
SNP: Single nucleotide polymorphism
